# Astroglial Connexins in Neurodegenerative Diseases

**DOI:** 10.3389/fnmol.2021.657514

**Published:** 2021-05-28

**Authors:** Xiaomin Huang, Yixun Su, Nan Wang, Hui Li, Zhigang Li, Guowei Yin, Hui Chen, Jianqin Niu, Chenju Yi

**Affiliations:** ^1^Research Centre, The Seventh Affiliated Hospital of Sun Yat-sen University, Shenzhen, China; ^2^School of Life Sciences, University of Technology Sydney, Sydney, NSW, Australia; ^3^Chongqing Key Laboratory of Neurobiology, Department of Histology and Embryology, Army Medical University (Third Military Medical University), Chongqing, China

**Keywords:** astrocyte, connexin, hemichannel, gap junction, neurodegenerative disease, Alzheimer’s disease

## Abstract

Astrocytes play a crucial role in the maintenance of the normal functions of the Central Nervous System (CNS). During the pathogenesis of neurodegenerative diseases, astrocytes undergo morphological and functional remodeling, a process called reactive astrogliosis, in response to the insults to the CNS. One of the key aspects of the reactive astrocytes is the change in the expression and function of connexins. Connexins are channel proteins that highly expressed in astrocytes, forming gap junction channels and hemichannels, allowing diffusional trafficking of small molecules. Alterations of astrocytic connexin expression and function found in neurodegenerative diseases have been shown to affect the disease progression by changing neuronal function and survival. In this review, we will summarize the role of astroglial connexins in neurodegenerative diseases including Alzheimer’s disease, Huntington’s disease, Parkinson’s disease, and amyotrophic lateral sclerosis. Also, we will discuss why targeting connexins can be a plausible therapeutic strategy to manage these neurodegenerative diseases.

## Introduction

Neurodegenerative diseases, presented as the progressive loss of structure or function of neurons, are the main threat to human health, especially for the geriatric population. The most common forms of neurodegenerative diseases include Alzheimer’s disease (AD), Parkinson’s disease (PD), Huntington’s disease (HD), amyotrophic lateral sclerosis (ALS) (Erkkinen et al., 2018). It is believed that different pathophysiological mechanisms causing these diseases are different and thus lead to different neurological outcomes. Some can cause memory and cognitive impairment (e.g., AD and PD), and others can affect people’s ability to move, speak, and breathe (e.g., PD, HD, and ALS) (Abeliovich and Gitler, 2016; Canter et al., 2016; Taylor et al., 2016; Wyss-Coray, 2016). However, treatment strategies which have been developed against the classical mechanisms are in-effective, yet treatments are urgently needed to stop or reverse the neurodegenerative diseases. This suggests that we may have missed some vital aspects in the bigger picture of neurodegenerative diseases.

For a long time, neuron-centered theories dominated the research interest of pathogenesis of neurological disorders, whereas the critical role of astrocytes in this process had been over-looked. In the last two decades, the role of astrocytes in the healthy and diseased brain started to gain some recognition. In the adult brain, astrocytes play several crucial roles in supporting neuronal functions, including forming the blood-brain barrier by interacting with endothelial cells, providing nutrients and metabolites support to neurons, and maintaining extracellular ion balance. These functions highly depend on the coordination of hundreds of astrocytes through the formation of an astrocytic network (Santello et al., 2019), which is crucial for cognition and other CNS function. The impairment of the astrocytic network has been found in neurodegenerative diseases (Cooper et al., 2020), where astrocytes undergo reactive gliosis with morphological and functional remodeling. Such changes have been suggested to contribute to the pathogenesis of neurodegenerative diseases (Pekny and Pekna, 2014).

The communication between astrocytes in the astrocytic network is achieved by sharing cytoplasmic content through specific membrane units called “gap junctions.” Gap junctions allow the transcellular exchange of ions and small molecules, such as Adenosine 5′-diphosphate, glucose, glutamate, glutathione, as well as secondary messengers including cAMP and inositol triphosphate. Connexin (Cx) is a protein family that forms the structural basis of gap junctions. Cx proteins are tetraspanins with two extracellular and one intracellular loop, while the NH_2_- and COOH-terminal tails are located in the intracellular space (Skerrett and Williams, 2017). Cx monomers are assembled into a hexamer connexon (also called “hemichannel”) on cell membranes, and two adjacently docked connexons in the neighboring cell membranes form gap junction channels (GJCs) (Figure 1). A cluster of GJCs composes the gap junction (Nielsen et al., 2012).

**FIGURE 1:** Connexin formation of hemichannel. **(A)** Connexin hexamer constitutes hemichannel, while hemichannels in the adjacent cells interact to form the gap junction channel. **(B)** Structure of Cx43 protein. Phosphorylation sites by MAPK, CK1, and PKC in the c-terminal tail are highlighted by white circles. Regions crucial for hemichannel activation regulation was also highlighted. **(C)** Proposed conformation changes that lead to hemichannel activation. Interaction of either CT9 or SH3-binding region with GAP19 region could achieve partial hemichannel activation, while interaction of both CT9 and SH3-binding region with GAP19 lead to fully activation of hemichannel (Iyyathurai et al., 2018). MAPK phosphorylation at S255, S262, S279, and S282 sites was proposed to facilitate interaction of SH3-binding region to the GAP19 region, enabling hemichannel activation (Freitas-Andrade et al., 2019). PKC phosphorylation at S386 could reduce the permeability of larger molecules such as sucrose (Bao et al., 2007; Hawat and Baroudi, 2008), which might act to interfere with the interaction between CT9 and GAP19 region. CK1 phosphorylation at S325, S328, and S330 has been shown to modulate hemichannel activity (Ek-Vitorín et al., 2018), but the mechanism is yet to be determined. ECM, extracellular matrix; MAPK, mitogen activated protein kinase; PKC, protein kinase C; CK1, casein kinase 1; SH3, SRC Homology 3; CT9, last 9 amino acids of the Cx43 C terminus; P labels phosphorylated amino acid residue.

During reactive gliosis, the expression and function of these Cx proteins changes in astrocytes (Giaume et al., 2010, 2021), especially the opening of Cx hemichannel. The opening of the hemichannel could be triggered in certain conditions, including lower pH, mechanical stimulation, oxidative stress, as well as inflammation caused by ischemic stroke and other injuries (Retamal et al., 2006, 2007; Sanchez et al., 2014; Turovsky et al., 2020). The opening of Cx hemichannels can release gliotransmitters including ATP, glutamate, and D-serine, to support normal neuronal function in the physiological situation (Meunier et al., 2017). However, overactivation of Cx hemichannels found in reactive astrogliosis during neurodegeneration has been shown to disrupt the microenvironment homeostasis and contribute to disease progression (Vis et al., 1998; Orellana et al., 2011b; Takeuchi et al., 2011; Wang et al., 2013; Almad et al., 2016; Yi et al., 2016; Maatouk et al., 2019).

In addition, the pannexin (Panx) protein family could also perform Cx-hemichannel-like activity (Yeung et al., 2020). Panx usually does not form GJCs (Sosinsky et al., 2011; Sahu et al., 2014) and Panx channels have similar membrane topology and pharmacological properties to Cx hemichannels. However, Panx and Cx exhibit no significant sequence homology (Yeung et al., 2020). Panx1 and Panx2 expression have been found in neurons, however, their expression in astrocytes is still controversial, which may depend on the pathological condition (Vogt et al., 2005; Yeung et al., 2020).

This review will focus on the current understanding of astrocytic Cx in neurodegenerative diseases, including AD, PD, HD, and ALS. We will examine how astroglial Cx, together with Panx, function as hemichannels and contribute toward the development of neurodegenerative diseases. Furthermore, we propose that astroglial hemichannels are potential therapeutic targets for the neurodegenerative diseases.

## Connexin Expression and Function in Astrocytes

In astrocytes, the dominant Cx proteins are Cx43 and Cx30, while Cx26 expression is also detectable (Rash et al.,2001a,b). Cx43 and Cx30 normally function as GJCs, as was repeatedly shown by experiments in acute brain slices from knockout mice, including the astrocytic Cx43 conditional knockout mice (hGFAP-cre:Cx43^*fl/fl*^), the Cx30 knockout mice (Dere et al., 2003; Theis et al., 2003), and the double KO mice (hGFAP-cre:Cx43^*fl/fl*^:Cx30 KO) (Wallraff et al., 2006; Rouach et al., 2008; Pannasch et al., 2011; Roux et al., 2011). The expression levels of these two Cxs in astrocytes varies in different brain regions (Batter et al., 1992; Nadarajah et al., 1996; Nagy et al., 1999), and can be changed in neurodegenerative diseases, such as AD (Mei et al., 2010; Yi et al., 2016; Angeli et al., 2020). Additionally, Cx26 has also been detected in certain astrocytes to a lesser extent (Altevogt and Paul, 2004; Lynn et al., 2011; Nagy et al., 2011). Panx1 was reported to be expressed and also contribute to hemichannel function in reactive astrocytes in disease models (Silverman et al., 2009; Karpuk et al., 2011; Santiago et al., 2011; Orellana et al., 2015; Yi et al., 2016; Maturana et al., 2017).

The CX43- and CX30-formed GJCs organize astrocytic networks with certain selectivity, which is crucial for normal neuronal function (Santello et al., 2019). For example, the astrocytic networks can coordinate the activities of local neuronal networks by transporting glutamate or glutamine (Giaume et al., 2010). In addition, the Cx30 and Cx43 mediated astrocytic networks can nourish distant neurons by mediating the delivery of glucose and lactic acid (Rouach et al., 2008; Clasadonte et al., 2017; Giaume et al., 2021). Cx30 and Cx43 are also present in the astrocyte endfeet which enwrap cerebral microvessels in honeycomb-like large sized puncta that helps to represent the end-feet boundaries. This structure provides a perivascular route to mediate the exchange between neighboring end-feet (Simard et al., 2003; Rouach et al., 2008; De Bock et al., 2017). Additionally, researchers found proliferative parenchymal cells in the hypothalamus in mice were decreased in conditional Cx30 and Cx43 knock out (Recabal et al., 2018), suggesting the potential of promoting neurogenesis by manipulating Cx30 and Cx43 function.

Normally, the permeability of Cx43 hemichannels is low under resting conditions (Contreras et al., 2003). They still act to modulate neuron synaptic function via the release of gliotransmitter, such as D-serine (Meunier et al., 2017). However, during reactive gliosis hemichannel permeability is dysregulated in a series of stress-associated conditions, such as inflammation (Orellana et al., 2009; De Bock et al., 2017), ischemia, oxidative stress (Ramachandran et al., 2007), or increased intracellular free Ca^2+^ concentration ([Ca^2+^]_*i*_) (De Vuyst et al., 2009). A recent study further revealed that the permeability of Cx43 hemichannels in astrocytes is modulated by cytokines and relies on the permeant species characters (Sáez et al., 2020). Furthermore, the interaction between Cx43 C-terminal tail and its cytoplasmic loop is critical for the hemichannel activity, which, in turn, can affect its GJC function (Iyyathurai et al., 2013). The SH3 binding domain and the last 9 amino acids of the C-terminal tail bind to the L2/GAP19 domain of the cytoplasmic loop, allowing full activation of hemichannels (Iyyathurai et al., 2018; Figure 1). This interaction might be regulated by phosphorylation at serine-residues in the C-terminal tail by kinases including mitogen-activated protein kinase (MAPK), protein kinase C (PKC), and casein kinase 1 (CK1) (Bao et al., 2007; Hawat and Baroudi, 2008; Ek-Vitorín et al., 2018; Freitas-Andrade et al., 2019; Figure 1). The suppression of Cx43 phosphorylation by CK1 delta can promote astrocyte survival and vascular regeneration in proliferative retinopathy (Slavi et al., 2018).

In addition, Panx1 expression has also been found in cultured astrocytes (Huang et al., 2007; Bianco et al., 2009; Iwabuchi and Kawahara, 2011), and the activation of the P2 × 7 receptor by BzATP induced ATP release through Panx1 hemichannels instead of Cx43 hemichannels (Iglesias et al., 2009). Nevertheless, the activation of Cx43 hemichannels but not Panx1 channels *in vitro* only occurs upon exposure to hypoxia-reoxygenation, pro-inflammatory cytokines, or amyloid-beta (Aβ) treatments (Froger et al., 2010; Orellana et al., 2010; Orellana et al., 2011b). Both Cx43 hemichannels and Panx1 channels were activated in fibroblast growth factor-treated astrocyte from the spinal cord (Garre et al., 2010), and in acute brain slices from a mouse abscess model (Karpuk et al., 2011). The astrocytic Panx1 channels were also found to be activated in the APP/PS1 familial AD mouse model (Yi et al., 2016).

## Astroglial Connexins in AD

AD is defined by progressive memory loss, behavioral deficits, and significant personality changes (Soria Lopez et al., 2019). Aβ plaques, neurofibrillary tangles, neuronal death, as well as synapse loss are characteristic features in AD brains. Notably, an invariant feature associated with Aβ plaques is reactive gliosis that includes activated microglia and reactive astrocytes (Nagele et al., 2004).

Twenty years ago, Nagy and colleagues have firstly demonstrated that astrocyte Cx43 protein levels are increased in the brain tissue of AD patients, especially around the Aβ plaques (Nagy et al., 1995), which has been repeatedly confirmed (Kajiwara et al., 2018), and is also found in the APP/PS1 mouse model (Mei et al., 2010; Yi et al., 2016). However, a recent study showed that the mRNA level of Cx43 is decreased in the cortex and thalamus area of another mouse model of AD, 5xFAD mice, albeit the increased protein levels (Angeli et al., 2020). Treatment of Aβ_25__–__35_ on primary astrocytes also results in a similar negative correlation between Cx43 mRNA and protein levels (Maulik et al., 2020). These pieces of evidence imply a possible unknown mechanism of Cx43 protein expression or turnover in AD pathology. Additionally, results from primary astrocyte culture suggested that Aβ_25__–__35_ does not alter *de novo* synthesized Cx43 membrane forward trafficking, but increases the internalization of Cx43, which may be responsible for the decreased GJC coupling and the increased hemichannel activity (Maulik et al., 2020).

The role of astrocytic Cxs functional alteration in AD has only been identified recently, revealing that the increased Cx HC opening in AD might contribute to neuronal dysfunction. Aβ aggregates and dense core Aβ plaques can induce reactive astrogliosis in AD patients and murine AD models (Nagele et al., 2004; Verkhratsky et al., 2010). The treatment of Aβ peptide in cultured astrocytes as well as in acute hippocampal slices has been shown to induce hemichannel opening, which releases glutamate and ATP, resulting in neuronal death (Orellana et al., 2011a). Similarly, in APP/PS1 mice, there is not only increased Cx43 and Cx30 expression in reactive astrocytes surrounding Aβ plaques, but also increased Cx43 hemichannel activity as shown in acute hippocampal slices; however, the GJC function was unaltered (Yi et al., 2016). Furthermore, conditional knockout of astrocytic Cx43 in APP/PS1 mice can block hemichannel activation and lead to reduced neuronal damage in the hippocampus (Yi et al., 2016). A more recent study has also shown that specific deletion of Cx43 in astrocytes ameliorates cognitive dysfunction in APP/PS1 mice (Ren et al., 2018). These studies confirmed a critical role of astrocytic Cx43 in causing neuronal damage in the AD model, suggesting that astrocytic Cx hemichannels function could be a possible therapeutic target of AD (Figure 2).

**FIGURE 2:** Schematic illustration of the role of astroglial hemichannels in neurodegeneration in an AD mouse model (APP/PS1). In the hippocampus, Cx43 HCs are activated in astrocytes contacting Aβ plaques which are triggered by high [Ca^2+^]_i_ ①, while Panx1 hemichannels are only activated as a minor contributor triggered by proinflammatory cytokines ② (Yi et al., 2016). HC opening results in the influx of Ca^2+^ from extracellular to cytoplasm, allowing the high [Ca^2+^]_*i*_ maintenance ③ (Yi et al., 2016). HCs activation in astrocytes can lead to gliotransmitter release including glutamate and ATP ④, which then stimulate the intracellular neurotoxic cascades and resulting in neurodegeneration ⑤ (Yi et al., 2016). The astroglial connexin hemichannel blockers [such as Boldine (Yi et al., 2017) and TAT-Gap19 (Abudara et al., 2014)] may become new pharmaceutical tools that can alleviate the neuronal damage in AD ⑥. AD, Alzheimer’s disease; HC, hemichannel; ECM, extracellular matrix.

Efforts have been made to screen or design compounds targeting astrocytic Cx proteins, in particular their hemichannel function, to ameliorate AD progression. It was reported that an alkaloid from the boldo tree called boldine could block the activation of hemichannels in astrocytes and microglia without affecting GJC both in cell culture and in acute hippocampal slices (Yi et al., 2017). In the AD murine model (APP/PS1), long-term oral administration of boldine could inhibit hemichannel activation in astrocytes, accompanied by reduced intracellular Ca^2+^ in astrocytes, decreased gliotransmitter release, and alleviated neuronal damage in the hippocampus (Yi et al., 2017). It was also found that endogenous and synthetic cannabinoid administration can reduce astrocyte Cx43 hemichannels activity and thereafter alleviate the neuronal damage in hippocampal slices exposed to Aβ (Gajardo-Gomez et al., 2017). However, more studies are required to confirm if pharmacological Cx hemichannel blockers could rescue cognitive function in AD, in order to pave the way for clinical applications.

## Astroglial Connexins in PD

PD, as the second most common neurodegenerative disease, is characterized by progressive dopaminergic neuronal loss in the striatum and substantia nigra (Beitz, 2014). The most characteristic hallmark of PD is Lewy bodies, which are cytoplasmic protein-based aggregations of α-synuclein. The clinical manifestations of PD include several motor dysfunction such as postural and movement disability, and non-motor symptoms including depression, psychosis, and dementia (Fernandez, 2012). Notably, astrogliosis in the substantia nigra plays a crucial role in PD pathogenesis (Cabezas et al., 2014).

The commonly used animal model of PD is 1-methyl-4-phenyl-1,2,3,6-tet- rahydropyridine (MPTP)-lesioned striatum which leads to neurodegeneration of dopaminergic neurons. In this PD model, the expression of Cx43 and Cx30 in the striatum is increased (Rufer et al., 1996; Fujita et al., 2018). A recent study showed that astrocytic Cx43 hemichannel permeability was also increased in the MPTP model, accompanied by elevated intracellular Ca^2+^ levels in the astrocytes of acute midbrain slices (Maatouk et al., 2019). The administration of a hemichannel inhibitor TAT-Gap19 peptide (Abudara et al., 2014), is able to rescue dopaminergic neuronal loss and inhibit microglial activation (Maatouk et al., 2019). These data suggest that astrocytic Cx hemichannel opening is detrimental to the neurons in the MPTP model. However, it appears that other aspects of astrocytic Cx function might be required for neuronal survival, as Cx30 KO enhanced the loss of dopaminergic neurons in MPTP treatment (Fujita et al., 2018). In Cx30 knockout mice receiving MPTP, reactive gliosis was suppressed and the expression of neuroprotective astrocytic genes was reduced, which may contribute to the exaggerated neuronal damage (Fujita et al., 2018). However, the exact function of Cx30 in the development of PD remained unknown. Rotenone, a mitochondrial complex I inhibitor, is another neurotoxic substance commonly used to generate rodent models of PD. Rotenone administration *in vivo* or *in vitro* can increase Cx43 protein level and its phosphorylation, and GJC function in astrocytes (Kawasaki et al., 2009).

Researchers also examined how α-synuclein affects astrocytic hemichannel function. It has been shown that α-synuclein also enhances the opening of Cx43 and Panx1 hemichannels in mouse cortical astrocytes, which results in the alterations in the intracellular Ca^2+^ dynamics, nitric oxide production, gliotransmitter release, mitochondrial morphology, and astrocyte survival (Díaz et al., 2019). This suggests that Cx43 and Panx 1 hemichannels may be involved in the pathogenesis of PD.

## Astroglial Connexins in HD and ALS

HD is characterized as a progressively autosomal-dominant neurodegenerative disorder, The features of HD include chorea, dystonia, cognition deficits, as well as behavioral impairments (Walker, 2007). In both healthy and diseased human brains, the distribution of Cx43 in the globus pallidus is homogeneously in the neuropil. However, in the caudate nucleus, the density of Cx43 is increased, which is formed in patches in HD. The immunoreactivity of the staining for glial fibrillary acidic protein (GFAP) in the astrocytes is also significantly higher in the caudate nucleus in HD brains compared to in healthy brains, and there is also increased reactive astrogliosis with elevated Cx43 expression associated with degenerating neurons (Vis et al., 1998). However, the contributions of Cx hemichannels in HD have been rarely reported in recent years and thus remain to be elucidated.

ALS is characterized by progressively weakened voluntary skeletal muscles, as well as those controlling swallowing, speech, and respiration (Oskarsson et al., 2018). It is a progressive and fatal neurodegenerative disease that occurs in the younger population compared with AD and PD. Cx43 expression was found to be upregulated in the motor cortex and spinal cord of patients with ALS and in a murine model of ALS (SOD1^*G*93A^) (Díaz-Amarilla et al., 2011; Almad et al., 2016). This upregulated Cx43 expression was accompanied by an increased hemichannel activity and gap junction coupling, and subsequently elevated concentration of intracellular Ca^2+^, which led to motor neuron damage. In addition, the administration of pan Cx43 blocker and Cx43 hemichannel inhibitors in the ALS mouse model can alleviate the neuronal toxicity (Takeuchi et al., 2011; Almad et al., 2016), suggesting that targeting Cx43 hemichannel function is a potential ALS treatment strategy. The upregulation of Panx1 expression is also found in the spinal cord of SOD1^*G*93A^ mice when the symptoms become apparent (Cunha et al., 2018). However, the role of Panx1 in ALS development has not been comprehensively studied, therefore its role is still unknown.

## Perspectives

The astrocytic GJCs and hemichannels formed by Cx proteins play important roles in neuroglial interactions. GJCs maintain neuronal homeostasis via astroglial and panglial networks for the trafficking of metabolic substances and elimination of potassium and glutamate. Under pathological conditions, the maintenance of GJC function may be beneficial as it is required for astrocytes to resist oxidative stress (Le et al., 2014). In contrast, while proper astroglial hemichannels opening is required for neuronal function under physiological conditions, hemichannel overactivation plays a detrimental role in several neurodegenerative disorders, such as AD, PD, and ALS.

Although it has been shown that Cx proteins could directly cause neuronal damage via hemichannel function in neurodegenerative diseases, they might also implicate in the disease pathogenesis by alternative mechanisms. Cx43 and Cx30 protein expression is enriched at the astrocyte endfeet at the gliovascular interface, and the absence of these astrocytic Cx proteins weakens the blood-brain barrier function (Ezan et al., 2012; Boulay et al., 2015), indicating a critical role of Cx proteins in the maintenance of the blood-brain barrier. Blood-brain barrier disruption has been found in neurodegenerative diseases including AD, PD, HD, and ALS (Sweeney et al., 2018; Huang et al., 2020). However, whether astrocytic Cx proteins contribute to these disease processes remains to be studied. In addition, astrocytic Cx proteins might also regulate the glymphatic pathway, which is constituted by the perivascular space wrapped by astrocytic endfeet and involved in protein waste clearance from the CNS (Rasmussen et al., 2018). Disruption of the glymphatic system has been identified in AD, which might hinder the export of Aβ protein (Nedergaard and Goldman, 2020). Considering the enrichment of Cx proteins at the astrocytic endfeet, they might also regulate glymphatic system function in neurodegenerative diseases.

Given their role in several neurodegenerative diseases, Cx and Panx hemichannels can be considered as promising alternative therapeutic targets. Hemichannels appear to be more associated with neurotoxicity compared to GJCs (Froger et al., 2010; Orellana et al., 2011a; Yi et al., 2016) and their cellular localizations enable pharmacological interventions. Indeed, several strategies using genetic or pharmacological tools to block hemichannel activity have been developed in recent years (Huang et al., 2012; O’Carroll et al., 2013; Bravo et al., 2014; Chen et al., 2014). Most of them inhibit the expression and/or function of Cx43, which is regarded as the major hemichannel component in astrocytes (Nagy et al., 2004). However, they also seem to impact astroglial GJC function, which results in an inaccurate interpretation of the findings. Therefore, a tool that can specifically block hemichannel function in glial cells may delineate the future direction that reduces potential off-target effects.

In neurodegenerative diseases, the development of a potential treatment must consider the needs of long-term treatment and also the use of molecules with the ability to cross the blood-brain-barrier. As such, boldine, an alkaloid compound as mentioned in earlier session, can block Cx43 hemichannels in astrocytes and microglia without affecting GJCs *in vitro* and in acute hippocampal slices from APP/PS1 mice at the age of 9 months (Yi et al., 2017). Three-month oral administration of boldine in APP/PS1 mice blocked the activation of astroglial hemichannels and ameliorated hippocampal neuritic dystrophies around the Aβ plaques (Yi et al., 2017). These results suggest that boldine seems to be a promising small molecule drug, which opens the revenue to design novel protective molecules that can alleviate neuronal toxicity under neurodegenerative conditions, especially the amyloid pathology. However, it needs to be noted that boldine has other functions, such as antioxidant and anti-inflammatory effects (Schulz et al., 2015), which can also participate in the protection of neurodegeneration in AD. Furthermore, several TAT-conjugated Cx43 peptidomimetics have been shown to block Cx43 hemichannel activity (Evans et al., 2012). For example, TAT-Gap19, a nonapeptide targeting on Cx43 extracellular loop, has been reported to exclusively block astroglial Cx43 hemichannel in a dose-dependent manner, without affecting GJCs (Abudara et al., 2014). Furthermore, in a mouse model of PD, TAT-Gap19 can protect against dopaminergic neuron degeneration and microglial activation (Maatouk et al., 2019). However, TAT peptides are susceptible to proteolytic cleavage in the blood (with a half-life less than 10 min, as determined by MALDI-TOF MS Analysis) (Grunwald et al., 2009), which limits its application in chronic diseases. Structural modification is needed to increase their half-life or slow down their release in the blood. More research is also needed to identify other inhibitors with high specificity to hemichannels and long half-life to enable later clinical translation.

## Conclusion

There is still a need for more in-depth investigations of astroglial Cx proteins, especially Cx43, in the pathology of neurodegenerative diseases not only in AD and PD but also in HD and ALS. Targeting astroglial Cx has become a potential strategy for the intervention or treatment of neurodegenerative diseases. Recent advances in the hemichannel opening mechanism have identified several regulatory regions in Cx43, which could facilitate the drug development targeting Cx hemichannel.

## Author Contributions

XH wrote the first draft of the manuscript. YS and HL revised the manuscript. NW, ZL, and GY edited the manuscript. HC, JN, and CY revised, edited, and supervised the manuscript. All authors contributed to the article and approved the submitted version.

## Conflict of Interest

The authors declare that the research was conducted in the absence of any commercial or financial relationships that could be construed as a potential conflict of interest.
